# MicroRNA-603 Promotes Progression of Cutaneous Melanoma by Regulating TBX5

**DOI:** 10.1155/2021/1888501

**Published:** 2021-12-31

**Authors:** Xianghua Dong, Ying Wang, Yan Qu, Junru Liu, Xien Feng, Xuechao Xu

**Affiliations:** ^1^Department of Dermatology, Yantai Municipal Laiyang Central Hospital, 265200, China; ^2^Mengyin County People's Hospital, Linyi, Shandong 276200, China; ^3^Department of Dermatology, Yantai Yuhuangding Hospital, Yantai 264010, China; ^4^Department of Dermatology, Yantai Yuhuangding Hospital Laishan Branch, Yantai 264010, China; ^5^Department of Dermatology, 970 Hospital of The PLA Joint Logistic Support Force, Yantai 264010, China

## Abstract

**Background:**

Although studies manifested that microRNA-603 plays a vital role in many cancers, the modulatory mechanism of microRNA-603 in cutaneous melanoma remains unknown. We aimed to investigate the roles of microRNA-603 in cutaneous melanoma cells.

**Methods:**

First, microRNA-603 expression in cutaneous melanoma cell lines was detected by qRT-PCR. The mRNA and protein expression levels of TBX5 in cutaneous melanoma cell lines were tested by qRT-PCR and western blot, respectively. In addition, the interaction between microRNA-603 and TBX5 was determined by dual-luciferase reporter gene assay, and their impacts on the growth of cutaneous melanoma cells were detected by cellular function experiments such as MTT, colony formation, and Transwell assays.

**Results:**

The expression level of microRNA-603 in human cutaneous melanoma cells was relatively upregulated. Overexpressing microRNA-603 could promote progression of cutaneous melanoma cells, while silencing microRNA-603 expression could suppress the malignant progression of cutaneous melanoma. In addition, TBX5 was lowly expressed in cutaneous melanoma cells. As confirmed by dual-luciferase assay, microRNA-603 could specifically bind to 3′UTR of TBX5 and regulate TBX5. The results of the rescue experiment demonstrated that inhibiting microRNA-603 expression could suppress the proliferation, migration, and invasion of cutaneous melanoma cells, but its suppressive effect could be restored by TBX5.

**Conclusion:**

MicroRNA-603 could regulate the expression of TBX5, thus promoting the malignant progression of cutaneous melanoma cells.

## 1. Introduction

MicroRNAs are a class of endogenous small noncoding RNA molecules, which play a negative role in regulating gene expression by binding to 3′ untranslated region (UTR) of the target mRNA to induce the translation inhibition or posttranscriptional degradation of mRNA [1, 2]. It is well known that the microRNA profiles in cancers vary from their profiles in the normal status, and dysregulated microRNAs affect tumor progress by microRNA-mRNA regulatory mechanisms [3]. MicroRNA-603 was identified as a tumor-promoting microRNA in several cancers. For instance, Guo et al.'s study [4] indicated that microRNA-603 activates tumor growth in the glioma cell. And in a study conducted by Ma et al. [5], it was explained that the microRNA-603/BRCC2 regulatory axis promotes osteosarcoma. However, for ovarian cancer, microRNA-603 is considered as a tumor suppressor [6]. Altogether, microRNA-603 seems to play diverse roles in cancers, so that much more extensive studies on microRNA-603 are urgently needed.

Cutaneous melanoma is a malignant skin cancer characterized by aggressive metastatic growth and poor prognosis [7]. Many studies reported the tumor promoting/suppressing mechanisms of microRNAs on melanoma. For example, several microRNAs, like microRNA-26a, microRNA-137, and microRNA-148, can serve as tumor suppressors by targeting MITF, a master regulatory gene, in melanoma [8–10], while some other microRNAs, like microRNA-10b, microRNA-17, and microRNA-19, are considered as tumor-promoting factors by targeting ITCH, ETV1, and PITX1, respectively, in melanoma [11–13]. Extensively, some researchers also focused on the effects of microRNAs on melanoma immunotherapy and drug resistance [14–16]. In conclusion, the microRNA-mRNA axis played a crucial role in melanoma development, therapy, and drug resistance; however, the microRNA-mRNA regulatory mechanisms in melanoma had not been fully understood.

In this study, microRNA-603 was exhibited to be remarkably overexpressed in human cutaneous melanoma cell lines, and it could promote progression of cutaneous melanoma cells. We further confirmed that the T-box transcription factor 5 (TBX5) was a direct regulatory target of microRNA-603. This study conducted an in-depth investigation on the expression levels of microRNA-603 and TBX5 in cutaneous melanoma and their influence on the development of melanoma cells. These studies provided a basis for new therapeutic targets of cutaneous melanoma.

## 2. Materials and Methods

### 2.1. Cell Lines and Cell Culture

Normal human melanocytes PIG1 (BNCC340321) and human cutaneous melanoma cell lines A375 (BNCC352140), M21 (BNCC340167), and SK-MEL-1 (BNCC342058) were all provided by the BeNa Culture Collection (BNCC). Human cutaneous melanoma cell lines WM35 (BFN60808633), Malme-3M (BFN607200871), and SK-MEL-30 (BFN60805921) were purchased from BLUFBIO (Shanghai) Biotechnology Development Co., Ltd.

PIG1, A375, and SK-MEL-1 cell lines were all incubated in RPMI-1640 medium containing 10% fetal bovine serum (FBS). Cell lines M21, WM35, Malme-3M, and SK-MEL-30 were cultivated in DMEM (Sigma, USA) plus 10% FBS (Hyclone; GE Healthcare Life Sciences, Logan, UT, USA). All cells were incubated in a constant temperature incubator at 37°C with 5% CO_2_.

### 2.2. Cell Transfection

Mimic NC, microRNA-603 mimic, inhibitor NC, microRNA-603 inhibitor, si-NC, and si-TBX5 were all designed by Sangon Biotech (Shanghai, China). Lipofectamine 2000 (Thermo Fisher Scientific, Inc.) was applied to transiently transfect the synthesized sequences or expression plasmids into human cutaneous melanoma cells Malme-3M and A375. Afterward, the cells were cultivated in a corresponding medium with 5% CO_2_ at 37°C for future use. Before transfection, all cells should be maintained in the complete medium for at least 24 h and be washed with phosphate-buffered saline (PBS, pH 7.4).

### 2.3. qRT-PCR

Total RNA was separated from the transfected cells with a TRIzol reagent (Life Technologies, Grand Island, NY, USA). RNA concentration was determined by NanoDrop 2000 System (Thermo Fisher Scientific, Inc., Waltham, MA, USA). According to kit instructions, microRNAs and mRNAs were reversely transcribed into cDNAs by miScript IIRT Kit (QIAGEN, USA) and PrimeScript RT Master Mix (TaKaRa, Dalian, China), respectively. Expression of microRNA-603 and TBX5 mRNA was measured by qRT-PCR with Applied Biosystems® 7500 Real-Time PCR Systems (Thermo Fisher Scientific, Waltham, MA) by using the SYBR® Premix Ex Taq™ II (TaKaRa Bio Inc., Shiga, Japan). U6 and GAPDH were served as internal references for microRNA-603 and TBX5, respectively. The 2^-*ΔΔ*Ct^ value was used to compare the difference between the relative expressions. Primer sequences are exhibited in Table 1.

### 2.4. Western Blot

After being washed twice with PBS, cells were lysed with radioimmunoprecipitation assay (RIPA) buffer (Thermo Fisher Scientific, MA, USA). Protein concentration was tested with a BCA (bicinchoninic acid) protein assay kit (Beyotime). Equivalent protein samples were isolated by 10% sodium dodecyl sulphate-polyacrylamide gel electrophoresis (50 *μ*g/lane). Then, the samples were transferred to a polyvinylidene fluoride or polyvinylidene difluoride membrane (ZY-160FP, Zeye Bio Co., Ltd., Shanghai, China). The membrane was arrested in 5% skimmed milk at 37°C for 2 h. Subsequently, it was washed 3 times with Tris-Buffered Saline and Tween 20 (TBST) and incubated overnight at 4°C with rabbit polyclonal antibody TBX5 (1 : 1000, ab259980, Abcam, Cambridge, UK). Rabbit polyclonal antibody GAPDH (1 : 2500, ab9485, Abcam, Cambridge, UK) was used as control. After being washed with TBST, the membrane was incubated with goat antirabbit IgG H&L (1 : 2000, ab205718, Abcam, Cambridge, UK) for 2 h. Finally, an enhanced chemiluminescent (ECL) kit (Pierce Biotechnology) was used to develop the membrane, and the protein bands were analyzed with an imaging system (ZG11SCIBRIGHTCL, Bio-Rad, CA, USA).

### 2.5. MTT Assay

After the melanoma cells Malme-3M and A375 were digested, centrifugated, and resuspended, 3 × 10^3^ cells were supplemented to each well of 96-well plates with three replicated wells and cultured under routine conditions. The cells were continuously cultured for 4 d, 10 *μ*L MTT was added for every 100 *μ*L culture medium every day, and the cells were incubated for 4 h. The absorbance values were measured at 570 nm by a microplate reader, and cell proliferation was evaluated. The cell growth curve was plotted with time being the horizontal axis and the absorbance ratio of cells in each group at each time point being the vertical axis.

### 2.6. Colony Formation Assay

After 48 h of transfection, 500 cells were placed on 6-well plates for cell culture. The culture mediums were replaced every 2 d. After culture for 15 d, the cells were washed twice with PBS, fixed with methanol at room temperature for 20 min, and stained with 0.1% crystal violet for 15 min. Finally, colonies with at least 50 cells were counted with a microscope.

### 2.7. Transwell Assay

*Cell migration assay*: 2 × 10^5^ transfected cells were inoculated into the upper chamber of a Transwell chamber, and a cell culture medium plus 10% FBS was added into the lower chamber to stimulate cell invasion. After culture for 24 h at 37°C, the inner and outer cells were gently removed. The remaining cells were fixed in 4% paraformaldehyde for 15 min and stained with 0.1% crystal violet for 20 min. The stained cells were observed by an optical microscope, and five regions were randomly selected at 100x magnification to calculate the number of stained cells. Then, statistical analysis was performed. Cell invasion detection was similar to cell migration assay except that cell invasion assay required a 20 *μ*g extracellular matrix gel (Sigma-Aldrich; Merck KGaA) being coated in the upper chamber.

### 2.8. Dual-Luciferase Assay

The synthesized mutant (MUT) or wild-type (WT) 3′UTR of TBX5 were cloned into the downstream of luciferase vector pmirGLO (Promega, WI, USA) to construct the luciferase reporter plasmids WT-TBX5 and MUT-TBX5. Subsequently, the human cutaneous melanoma cells Malme-3M were cotransfected with the plasmids and microRNA-603 mimic or mimic NC, while A375 cells were cotransfected with the plasmids and microRNA-603 inhibitor or inhibitor NC. Renilla luciferase expression vector pRL-TK (TaKaRa, Dalian, China) was used as internal reference. The luciferase activity was tested by a dual-luciferase assay kit (Promega, Madison, WI, USA).

### 2.9. Data Analysis

The experimental data were analyzed by GraphPad Prism 6.0 software (GraphPad Prism 6.0, San Diego, CA, USA). The above cell experiments were all repeated three times. The measurement data were expressed as mean ± standard deviation. The comparison between the two groups was examined by Student's *t*-test. *p* < 0.05 refers to statistically significant differences.

## 3. Results

### 3.1. MicroRNA-603 Expression Is Significantly Elevated in Different Melanoma Cell Lines

As studies showed, microRNA-603 is generally fostered in a variety of cancer tissues and usually stabilizes the development of tumors, like osteosarcoma [5], glioma [4], and colorectal cancer [17]. Here, we tested microRNA-603 expression via qRT-PCR. The results unveiled that microRNA-603 in human cutaneous melanoma cell lines was higher than that in the normal human melanoma cell line (Figure 1). Therefore, melanoma cells Malme-3M with the lowest microRNA-603 expression level and A375 with the highest microRNA-603 expression level were selected for subsequent cellular function experiments.

### 3.2. Overexpressing MicroRNA-603 Promotes Progression of Melanoma Cells Malme-3M

To explore the biological functions of microRNA-603 in melanoma cells, mimic NC and microRNA-603 mimic were transfected into melanoma cells Malme-3M. After transfection and culture for 2 d, the microRNA-603 level was measured by qRT-PCR. The result indicated that the microRNA-603 overexpression could effectively increase the expression of microRNA-603 (Figure 2(a)). Then, the result of MTT assay suggested that the proliferative ability of melanoma cells in overexpressing microRNA-603 group was stronger (Figure 2(b)). Moreover, clonality of melanoma cells transfected with the microRNA-603 mimic was also notably enhanced (Figure 2(c)). Transwell assay results are shown in Figures 2(d) and 2(e). In comparison with the negative control group, cell migratory and invasive abilities in the microRNA-603 mimic group were enhanced. In conclusion, upregulation of microRNA-603 could facilitate the malignant process of melanoma cells.

### 3.3. Downregulation of MicroRNA-603 Inhibits Progression of Melanoma Cells

Similarly, inhibitor NC and the microRNA-603 inhibitor were utilized to transfect melanoma cells A375. After 2 d of transfection and culture, the qRT-PCR result suggested that in the microRNA-603 inhibitor experimental group, the expression level of microRNA-603 was lower than that in the control group (Figure 3(a)). Thus, the transfected cells could be utilized for subsequent experiments. Next, as exhibited in Figures 3(b) and 3(c), compared with negative control group, the proliferative ability and clonality of melanoma cells were both inhibited in the microRNA-603 inhibitor experimental group. Transwell assay results were demonstrated in Figures 3(d) and 3(e). Compared with the negative control group, cell migratory and invasive abilities of the microRNA-603 inhibitor group were both attenuated. Hence, we assumed that silencing microRNA-603 could inhibit the progression of melanoma cells. Concluding the results from the Sections 2.2 and 2.3, microRNA-603 could affect proliferation, migration, and invasion of cutaneous melanoma cells.

### 3.4. TBX5 Expression Is Downregulated in Melanoma Cells and Is a Direct Regulatory Target of MicroRNA-603

To better understand the molecular mechanisms of microRNA-603 affecting the phenotype of melanoma cells, the downstream regulatory axis was explored. As the literature review illustrated, TBX5 is a tumor suppressor and can be downregulated by some oncomicroRNAs [18, 19]. Therefore, we assumed that microRNA-603 could bind to TBX5 mRNA, thus suppressing its expression at a posttranscriptional level. To identify the binding relationship, the TargetScan database was applied to predict the binding site between microRNA-603 and TBX5, and the results verified this binding relationship (Figure 4(a)). Synthesized MUT or WT 3′UTR of TBX5 was cloned into the downstream of the pmirGLO luciferase vector, so as to construct luciferase reporter plasmids TBX5-WT and TBX5-MUT (Figure 4(b)). First, qRT-PCR and western blot results manifested that compared with the normal human melanocyte cell line, TBX5 expression in melanomas was downregulated (Figure 4(c)). Next, dual-luciferase reporter gene assays confirmed that cotransfecting TBX5-WT with the microRNA-603 mimic or the microRNA-603 inhibitor could induce decreased or increased luciferase activities, respectively, while no luciferase activity changed in the transfection group using TBX5-MUT (Figure 4(d)). Additionally, qRT-PCR and western blot assays also demonstrated that transfection of the microRNA-603 mimic could significantly reduce the expression of TBX5 in Malme-3M cells, while transfection of the microRNA-603 inhibitor could notably increase the expression of TBX5 in A375 cells (Figures 4(e) and 4(f)). These results suggested that microRNA-603 could downregulate the TBX5 expression by directly targeting it.

### 3.5. MicroRNA-603 Affects Progression of Melanoma Cells by Regulating TBX5

We confirmed that in melanoma cell lines, microRNA-603 was highly expressed. Then, in order to better verify the correlation between microRNA-603 and TBX5 as well as their effects on melanoma cell behaviors, a series of cellular function experiments were conducted. Firstly, transfection groups of the melanoma cell line A375 were constructed, including the inhibitor NC+si-NC, microRNA-603 inhibitor+si-NC, and microRNA-603 inhibitor+si-TBX5 groups. qRT-PCR and western blot results are exhibited in Figure 5(a). Compared with the control group, the TBX5 expression was elevated when the microRNA-603 expression was suppressed, while the expression of TBX5 was inhibited when the two genes were silenced simultaneously. In MTT and the colony formation assay, it was observed that the proliferative activity and clonality of cancer cells were both decreased in A375 cells transfected with the microRNA-603 inhibitor. Nevertheless, when microRNA-603 and TBX5 were inhibited simultaneously, the proliferative ability of the cells was notably restored (Figures 5(b) and 5(c)). In addition, Transwell assay results were demonstrated in Figures 5(d) and 5(e). Compared with the negative control group, cell migratory and invasive abilities were both suppressed in the microRNA-603 inhibitor+si-NC group. However, in the microRNA-603 inhibitor+si-TBX5 transfection group, the migratory and invasive abilities of cancer cells were significantly restored. Therefore, these results jointly suggested that lowly expressed microRNA-603 could suppress the proliferation, migration, and invasion of melanoma cells, while its inhibitory effect could be offset by silencing TBX5.

## 4. Discussion

In this study, we first examined microRNA-603 in cutaneous melanoma cell lines through qRT-PCR. Experimental results demonstrated that the microRNA-603 expression in cutaneous melanoma cell lines was generally higher than that in normal tissue. To explore the effect of microRNA-603 on the changes of cellular functions of cutaneous melanoma cells, microRNA-603 was overexpressed and suppressed in cutaneous melanoma cell lines Malme-3M and A375, respectively, so as to observe the changes in cell proliferation, migration, and invasion, etc. The results illustrated that microRNA-603 facilitated proliferation, migration, and invasion of cutaneous melanoma cells, which revealed that microRNA-603 was very likely to act as a cancer-promoting factor in cutaneous melanoma.

TBX5 is a member of a phylogenetic conserved gene family. This family shares the same DNA binding domain known as T-box. TBX5 containing T-box sequence can be utilized as a transcription factor to induce apoptosis, inhibit cell proliferation [20] and intercellular signal transduction [21], and negatively modulate cell migration by regulating transcription [22]. Studies confirmed that TBX5 plays a part in suppressing cancer in a variety of cancer tissues. For instance, in colon cancer [23], TBX5 has a high degree of methylation and a low expression level. TBX5 is generally low in nonsmall cell lung cancer, and upregulation of TBX5 markedly represses progression of cancer cells [18]. Nevertheless, the molecular modulatory mechanism of TBX5 in melanoma remains unclear. Therefore, we selected it as our research object, and we predicted the binding site between TBX5 and microRNA-603 through the TargetScan database. Then, the dual-luciferase assay was performed to verify that TBX5 was the direct regulatory target of microRNA-603. TBX5 was downregulated in cutaneous melanoma cells, and its expression level was modulated by microRNA-603. Based on the expression status of microRNA-603 and TBX5, and the binding interaction between them, we proposed the microRNA-603/TBX5 axis in cutaneous melanoma.

In summary, in this study, it was manifested that microRNA-603 was remarkably upregulated in cutaneous melanoma cells, and it played a role as a cancer-promoting factor by targeting and regulating TBX5 expression. This study is helpful for the understanding of the biological functions of the microRNA-603/TBX5 regulatory axis in the occurrence of tumors, which is expected to offer a new target for the molecular therapy of cutaneous melanoma.

## Figures and Tables

**Figure 1:** MicroRNA-603 expression is notably upregulated in different melanoma cell lines. Expression of microRNA-603 in normal human melanocyte cell line PIG1 and different melanoma cell lines (A375, M21, SK-MEL-1, WM35, Malme-3M, and SK-MEL-30). ∗ indicates *p* < 0.05.

**Figure 2:** Overexpressing microRNA-603 promotes progression of melanoma cells Malme-3M. (a) Expression level of microRNA-603 after melanoma cell line Malme-3M transfected with mimic NC and microRNA-603 mimic; (b) the proliferative ability of melanoma cells Malme-3M in overexpressed microRNA-603 group and control group; (c) clonality of melanoma cells Malme-3M in overexpressed microRNA-603 group and control group; (d) migratory ability of melanoma cells Malme-3M in overexpressed microRNA-603 group and control group (100x); (e) invasive ability of melanoma cells Malme-3M in overexpressed microRNA-603 group and control group (100x). ∗ indicates *p* < 0.05.

**Figure 3:** Lowly expressed microRNA-603 inhibits proliferation, migration, and invasion of melanoma cells. (a) Expression level of microRNA-603 after melanoma cell line A375 was transfected with inhibitor NC and microRNA-603 inhibitor; (b) proliferative ability of melanoma cells A375 in microRNA-603 inhibitor experimental group and control group; (c) clonality of melanoma cells A375 in microRNA-603 inhibitor experimental group and control group; (d) migratory ability of melanoma cells A375in microRNA-603 inhibitor experimental group and control group (100x); (e) invasive ability of melanoma cells A375 in microRNA-603 inhibitor experimental group and control group (100x). ∗ indicates *p* < 0.05.

**Figure 4:** TBX5 is less expressed in melanoma cells and is a direct regulatory target of microRNA-603. (a) The targeting binding site of microRNA-603 and TBX5 3′UTR; (b) schematic diagram of luciferase reporter plasmids TBX5-WT and TBX5-MUT; (c) the mRNA and protein expression levels of TBX5 in human normal melanocyte cell line PIG1 and melanoma cell lines Malme-3M and A375; (d) the targeted binding of microRNA-603 and TBX5; (e) the effect of abnormal expression level of microRNA-603 on the mRNA expression of TBX5; (f) the influence of abnormal expression level of microRNA-603 on protein expression of TBX5. ∗ means *p* < 0.05.

**Figure 5:** MicroRNA-603 affects progression of melanoma cells by regulating TBX5. (a) The mRNA and protein expression levels of TBX5 in transfected cell line A375; (b) proliferative ability of cells in each transfection group of human cutaneous melanoma cell line A375; (c) clonality of cells in each transfection group of human cutaneous melanoma cell line A375; (d, e) migratory and invasive abilities in each transfection group of human cutaneous melanoma cell line A375 (100x). ∗ indicates *p* < 0.05.

**Table 1:** qRT-PCR primer sequences.

Genes	Primer sequences (5′-3′)
miR-603	F: CACACACUGCAAUUACUUUUGC

U6	F: CTCGCTTCGGCAGCACA
	R: AACGCTTCACGAATTTGCGT

TBX5	F: CTGTGGCTAAAATTCCACGAAGT
	R: GTGATCGTCGGCAGGTACAAT

GAPDH	F: GGAGCGAGATCCCTCCAAAAT
	R: GGCTGTTGTCATACTTCTCATGG

## Data Availability

The data used to support the findings of this study are available from the corresponding author upon request.
